# Genome-wide analysis of sucrose synthase family in soybean and their expression in response to abiotic stress and seed development

**DOI:** 10.1371/journal.pone.0264269

**Published:** 2022-02-25

**Authors:** Muhammad Zulfiqar Ahmad, Hafiz Ishfaq Ahmad, Asma Gul, Zamarud Shah, Bushra Ahmad, Shakeel Ahmed, Abdullah Ahmed Al-Ghamdi, Mohamed S. Elshikh, Arshad Jamil, Jamal Abdul Nasir, Helena Dvořáčková, Jan Dvořáček

**Affiliations:** 1 Department of Plant Breeding and Genetics, University of Agriculture, D.I. Khan, Pakistan; 2 Department of Animal Breeding and Genetics, University of Veterinary and Animal Sciences, Lahore, Pakistan; 3 Department of Statistics, Shaheed Benazir Bhutto Women University, Peshawar, Pakistan; 4 Department of Biotechnology, University of Science and Technology, Bannu, Pakistan; 5 Department of Biochemistry, Shaheed Benazir Bhutto Women University, Peshawar, Pakistan; 6 Institute de Farmacia, Facultad de Ciencias, Universidad Austral de Chile, Campus Isla Teja, Valdivia, Chile; 7 Department of Botany and Microbiology, College of Science, King Saud University, Riyadh, Saudi Arabia; 8 Department of Plant Breeding and Genetics, Gomal University, D.I. Khan, Pakistan; 9 Department of Agrochemistry, Soil Science, Microbiology and Plant Nutrition, Faculty of AgriSciences, Mendel University in Brno, Brno, Czech Republic; 10 Pedologiejh, spol s.r.o, Brno, Czech Republic; Ghazi University Dera Ghazi Khan, PAKISTAN

## Abstract

The sucrose synthase (SS) is an important enzyme family which play a vital role in sugar metabolism to improve the fruit quality of the plants. In many plant species, the members of SS family have been investigated but the detailed information is not available in legumes particularly and *Glycine max* specifically. In the present study, we found thirteen SS members (GmSS1-GmSS13) in *G*. *max* genome. High conserved regions were present in the GmSS sequences that may due to the selection pressure during evolutionary events. The segmental duplication was the major factor to increase the number of GmSS family members. The identified thirteen *GmSS* genes were divided into Class I, Class II and Class III with variable numbers of genes in each class. The protein interaction of GmSS gave the co-expression of sucrose synthase with glucose-1-phosphate adenylyltransferase while SLAC and REL test found number of positive sites in the coding sequences of SS family members. All the GmSS family members except *GmSS7* and few of class III members, were highly expressed in all the soybean tissues. The expression of the class I members decreased during seed development, whireas, the class II members expression increased during the seed developing, may involve in sugar metabolism during seed development. Solexa sequencing libraries of acidic condition (pH 4.2) stress samples showed that the expression of class I GmSS genes increased 1- to 2-folds in treated samples than control. The differential expression pattern was observed between the members of a paralogous. This study provides detailed genome-wide analysis of GmSS family in soybean that will provide new insights for future evolutionary and soybean breeding to improve the plant growth and development.

## Introduction

Sucrose is the key photosynthesis product that used in the cellular metabolism of higher plants. Number of metabolic pathways start from the breakdown of sucrose within the plant tissues. Sucrose synthases or invertases were responsible for the cleavage of sucrose [1]. The sucrose and uridine diphosphate was used as precursor for SS to convert them into fructose and UDP-glucose and can also catalyze the reversible reaction [2, 3]. SS family members also had vital metabolic function in plant growth and development processes. SS function normally suggested to use the UDP-glucose as substrate to synthesized the cellulose, that is vital for cell wall thickening and fiber cell development in cotton [4–6]. The SS genes also take part in starch storage in different crops organs like tubers, different root vegetables, kernels and pea embryos [7–10], import of sugar [11, 12], response to different environmental stresses [13, 14] and also involved in nitrogen fixation, arbuscule maintenance and maturation in mycorrhizal legume roots [15, 16]. The SS genes performed a wide range of function in the plant species and expressed distinctly in different tissues. The maize three SS genes expressed highly in developing kernels [17] but *Sh1* performed central role in cell wall synthesis while *Sus1* involved in starch synthesis [18]. The Pea *Sus1* was universally highly expressed in different seed developing stages, *Sus2* in old leaves and testas while low or weak expression of *Sus3* was observed in flower and young testas. Additionally, Pea *Sus1* genes activity was not found in mutant seeds while the expression was not compensated the *Sus2* and *Sus3* in root nodules [7].

Soybean, one of the leading legume crop, is much sensitive to low pH stress conditions that have great impact on its growth and yield [19]. Very little is known about legumes is general and soybean in specific response and tolerance mechanism against low pH and Al stresses conditions, may be due to their large genomes size, complex genetics and intricate resistance mechanism [19, 20]. Sucrose synthases predicted to have role in plant tolerance against Al stress because its transcript was significantly increased under combine effect of low pH (4.0)+Al+ PEG than control barley plants [21]. In view of SS genes importance and diverse functions in response to H^+^ and Al^3+^ phytotoxicity, Solexa sequencing libraries were used to study the GmSS genes response to low pH tolerance.

The whole Genome sequence of different crops open the gate of mining the respective gene family and their characterization. Similarly, adopting the genome-wide approach, six SS family members were reported in model legume plant, *Lotus japonicas* L [22], three SS genes were identified and characterized in rice [23, 24], six in *A*. *thaliana* and recently, five SS genes was identified in grapevine [25]. Zhu et al. 2017 also mentioned the eleven *G*. *max* SS genes but we find 13 SS family members in *G*. *max*. The Whole-Genome sequencing revealed to investigate the soybean SS gene family more thoroughly.

Soybean is not only the most important legume crop of the world but also present the key place for oil purpose. The identification and expression pattern analysis of all the members of a gene family is very important to understand the fully molecular biology and evolutionary study. In this study, we have identified the 13 SS family members in soybean and their transcript expression was investigated. The results of present study will provide the gateway to investigate and understand the possible role of SS enzymes in soybean plants, especially during the different developmental stages of the soybean crop.

## Materials and methods

### Sucrose synthase family genes identification in soybean

The online database, Phytozome 11.0 [26] and Soykb (http://soykb.org; [27]) was used to mine the SS genes from soybean genome by using Arabidopsis SS protein (AT1G73370) sequence as a query. The NCBI database (https://www.ncbi.nlm.nih.gov/Structure/cdd/wrpsb.cgi; [28]) was used to find out the conserved domain (PF00862) and discarded the SS domain lacking genes. The presence of SS specific domain was also confirmed in the non-redundant SS protein sequences through pfam and finally got the 13 GmSS genes. The genomics, CDS and 1.5 kbp upstream promoter region of the confirmed genes was extracted from soybean genome by using online database, Phytozome 11.0 [26] and Soykb (http://soykb.org; [27]).

### Physical properties, position on chromosome and sequence alignment

The physical properties of GmSS genes like number of amino acid, start-end position of the gene, chromosome location of GmSS family was taken from Phytozome. The molecular weight (kDs) and isoelectric point (pI) was calculated in the ExPASy tools (http://www.expasy.org/tools; [29]) with standard parameters by using the protein sequence of respective gene. The PhenoGram Plot (http://visualization.ritchielab.psu.edu/phenograms/plot; [30]) was used to show the GmSS genes on their respective chromosome. In MEGA 7.0 [31], ClustalW was used to align the amino acid sequence of GmSS and was applied to the GeneDoc tool to shade the conserved amino acids in alignment [32].

### Phylogenetic relationship, motifs and promoter region analysis

MEGA 7.0 [31] was used to construct the phylogenetic tree among GmSS, AtSS and other crop plants candidate genes by using neighbor joining method with bootstrap test involving 1000 replicates. The conserved region within GmSS genes were executed through MEME (http://memesuite.org; [33]) and their genomic assemblies were screened through Pfam database (http://pfam.sanger.ac.uk; [34]). The Plant cis-acting Regulatory DNA Elements (PlantCARE) program (http://bioinformatics.psb.ugent.be/webtools/plantcare; [35]) was used to analyse the 1.5kb upstream promoter region of each GmSS gene.

### Gene duplication, Ka/Ks calculation and positive selection analysis

The selection mode of each GmSS paralogous pair was evaluated by calculating the synonymous (Ks), non-synonymous (Ka) substitution rate and their ratio through online tool (http://services.cbu.uib.no/tools/kaks). The positive, purifying or neutral selection pressure of each duplicated GmSS gene was evaluated through Ka/Ks ratio. The Ka/Ks ratio > 1, < 1 or = 1 indicates the positive, purifying or neutral selection, respectively. The T = Ks/2λ formula (λ = 6.161029 x 10^−9^) was used to calculate the divergence time (T) of each GmSS pair [36]. The amino acid under selection pressure within the GmSS proteins was further confirmed through Selecton 2.2 (http://selecton.tau.ac.il; [37, 38]). Maximum-likelihood test through Bayesian inference methods was used to measure the shifted ω ratio between codons within the aligned sequences [39, 40]. The amino acids under the positive, neutral and purifying selections were appeared in the Selecton results and evaluated through scale color.

### Positive selection analysis on the basis of codon

Different likelihood approaches like random effect likelihood (REL), and single likelihood ancestor counting (SLAC) were used in online tool DATAMONKEY (http://classic.datamonkey.org/; [41–43]) by using coding sequence of SS genes to identify the positive sites through synonymous and non-synonymous variant calculation at each site by ω values.

### Synteny analysis

Genome fasta and general feature format (GFF) files of *G*. *max* and *A*. *thaliana* were extracted from online database phytozome. The files were subjected to One Step MCScan to determine the “syntenic genes” were used for synteny analysis. Dual Systeny Plot in TBTool [44] was used to display orthologous of SS genes located on syntenic chromosome blocks.

### Analysis of protein-protein interaction (PPI) network

The STRING version 9.1 (http://www.string-db.org; [45]) was used to determine the GmSS5 PPI network to understand their functioning mechanism at molecular level [46]. The PPI was sought out by using cutoff standard in the pooled score < 4. In the PPI network, the biological important and vastly interacted protein was placed in the central node by calculating the middle value and different lines were used to connect with different interacted proteins.

### In sillico expression analysis

The moicroarray transcript level expression data of identified GmSS genes in seven tissue (Seed, Root, Nodule, Stem, Leaf, Flower, Pod; S2 Table in S1 File) was obtained from phytozome 12.0 database (https://phytozome.jgi.doe.gov/pz/portal.html; [47]) and analysed for their transcript level expression.

Transcriptomic/expression data of soybean seed development was extracted from relevant literature (GSE79327) using NCBI GEO database. Transcriptomic profile of Dongnong47 (DN47) cultivar were compared using Illumina high-throughput RNA-sequencing on samples at 25, 35, 50, and 55 days after flowering (DAF). Seeds at 18 DAF served as the control [48].

Transcriptomic/expression data of soybean response to low pH was extracted from relevant literature (GSE129320) using NCBI GEO database. Transcriptome analyses of soybean roots response to acidity stress were carried out using pH4.2 as acid treatment and pH5.8 as control with three replicates [49].

## Results

### Characteristics of soybean SS gene family

Eleven SS family members from soybean genome were mentioned previously [25] and we have verified and replenished another two soybean SS genes (*Glyma11g33240* and *Glyma18g04990*) from *G*. *max* genome. These two new genes were named as *GmSS12* and *GmSS13*. Finally, thirteen non-redundant SS genes were investigated and analysed. Slightly variation in the properties of SS genes were observed between our and Zhu et al. [25] study with respect to DNA length and amino acid numbers. These thirteen SS genes were names as *GmSS1-GmSS13* and their physical properties were elaborated in Table 1. The size of GmSS genes were varied from 2238 (*GmSS13*) to 2766 (*GmSS4*) bp. The full length polypeptide through molecular analysis showed that predicted GmSS proteins contains 746 to 922 amino acids with predicted molecular weight of 84.76 kDs to 104.15 kDs. The pI ranged from acidic 5.76 (GmSS2) to basic 7.57 (GmSS13) (Table 1). The variation in the properties of GmSS genes indicates their diverse role in various microenvironments. All the GmSS genes were predicted to subcellularily localized in cytoplasm of the cell (Table 1).

**Table 1:** Properties of thirteen GmSS genes.

Class	Glyma ID	Gene Name	Start	End	CDS (bp)	Protein (A.A)	Protein (kDs)	pI	Localization
Class I	Glyma09g08550	GmSS3	7845478	7851685	2433	811	93.66	6.02	Cyto
	Glyma15g20180	GmSS8	17937869	17944091	2421	807	92.72	5.87	Cyto
	Glyma13g17421	GmSS5	21211872	21217120	2418	806	92.24	6.04	Cyto
	Glyma17g05067	GmSS10	3412682	3418160	2418	806	92.19	5.93	Cyto
Class II	Glyma15g16171	GmSS7	12475953	12483800	2409	803	91.57	5.84	Cyto
	Glyma03g37441	GmSS2	44041487	44047783	2439	813	92.31	5.76	Cyto
	Glyma19g40041	GmSS11	46515393	46521627	2439	813	92.26	5.95	Cyto
Class III	Glyma09g29710	GmSS4	36530532	36536435	2766	922	104.15	6.61	Cyto
	Glyma16g34290	GmSS9	36921331	36926993	2763	921	103.91	6.66	Cyto
	Glyma02g40740	GmSS1	45967536	45973138	2523	841	95.33	6.81	Cyto
	Glyma14g39070	GmSS6	48197559	48203317	2523	841	95.28	7.02	Cyto
	Glyma11g33240	GmSS12	30547238	30552421	2538	846	95.77	6.53	Cyto
	Glyma18g04990	GmSS13	3718552	3722900	2238	746	84.76	7.57	Cyto/Mit

The genes were arranged according to their placement in different classes.

Cyto: Cytoplasm.

Mit: Mitochondria.

Moreover, except in GmSS12 and GmSS13, conserved Ser residues were found at N-terminal regions of all the GmSS amino acid sequences (Fig 1), that related to the phosporylation in maize and cotton [50–52]. These typical signatures of SS proteins residues were also found in the GmSS genes (Fig 1). The different GmSS gene encodes different isoenzymes that have important function in soybean sucrose synthasis.

**Fig 1:** Predicted amino acid sequences of thirteen *GmSS* genes. Amino acid sequence alignment of 13 GmSS proteins was done with MEGA7. MEGA7 alignment was used in GeneDoc program to shade the identical and similar amino acids in alignment. The conserved serine residue for phosphorylation by Ser/Thr protein kinase is showed by an arrow-head. The characteristic sucrose synthase domain (broken underline) and a glycosyl transferases domain (single underline) were identified by the Interproscan algorithm (http://www.ebi.ac.uk/Tools/pfa/iprscan/). Dark shad represents identical amino acids and grey shade indicates similar amino acids.

Multiple sequence alignment analysis showed the high rang of similarities within the GmSS genes. The GmSS1 and GmSS6 shares 97.5% sequence similarity at amino acid level and found to be more closely related paralogous. Whereas, GmSS2 with GmSS11, GmSS3 with GmSS8, GmSS4 with GmSS9, GmSS5 with GmSS10 shares more than 90% identity at protein level (Table 2). The GmSS13 shares less identity and similarity with all the other GmSS genes at protein level (Table 2).

**Table 2:** Similarities and identities among thirteen GmSS genes.

	GmSS1	GmSS2	GmSS3	GmSS4	GmSS5	GmSS6	GmSS7	GmSS8	GmSS9	GmSS10	GmSS11	GmSS12	GmSS13
**GmSS1**		53.51	51.67	64.39	52.5	97.5	51.79	51.9	64.78	52.62	54.22	81.78	66.83
**GmSS2**	68.1		69.9	48.53	70.94	53.63	74.75	70.81	48.48	70.57	97.04	52.01	46.38
**GmSS3**	67.14	80.22		46.69	88.4	51.55	66.17	97.28	46.96	87.53	69.41	49.82	44.61
**GmSS4**	74.92	61.35	60.04		47.88	64.6	46.69	47.01	95.98	48.21	48.43	62.58	51.61
**GmSS5**	67.86	81.03	92.72	60.8		52.74	92	90.07	48.26	98.88	70.69	51.12	45.75
**GmSS6**	98.45	67.9	66.79	75.14	67.86		51.79	51.79	64.89	52.86	54.34	81.89	66.83
**GmSS7**	65.83	85.22	77.86	59.83	78.96	65.71		66.5	47.17	67.45	75	51.12	45.62
**GmSS8**	67.74	81.28	97.78	60.48	94.17	67.38	78.99		47.28	89.21	70.32	50.3	44.83
**GmSS9**	75.11	61.41	60.11	97.18	60.87	75.54	60.11	60.54		48.59	48.48	63.3	52.23
**GmSS10**	67.98	80.79	92.47	60.8	99.63	67.98	78.71	93.82	60.87		70.32	51.24	45.62
**GmSS11**	68.85	98.52	80.34	61.67	81.16	68.73	85.22	81.4	61.85	80.91		52.6	46.87
**GmSS12**	87.69	65.72	64.26	72.99	65.44	87.81	64.5	64.85	73.18	65.44	66.43		75.98
**GmSS13**	72.53	59.26	57.48	61.5	58.69	72.77	58.08	57.76	61.67	58.69	59.63	78.7	

Upper values showing identity (%) and lower values showing similarity (%) at protein level.

### Chromosome localization, duplication and evolutionary analysis of GmSS

The chromosomal positioning and GmSS genes initiation sites were specified by constructing chromosomal location map (Fig 2). Among the 20 soybean chromosomes, only 11 contains the thirteen SS genes. Two GmSS were located on each chromosome 9 and 15 while other chromosomes contains only 1 GmSS gene (Fig 2). Such SS genes distribution pattern was also observed in Cotton, Grapevine and Arabidopsis [25, 53].

**Fig 2:** Chromosomal locations and duplications of soybean SS genes. The chromosome number is indicated above each bar. The chromosome size is indicated by its relative length using the information from Phytozome and SoyBase. Each pair of segmental duplication is indicated by a rline of espective class color.

The gene duplication play an important role in the gene family extension and variation in their functions [54]. There were three main events i.e., segmental, tandem or whole genome through which the genome duplication event occurred in an organism. An ancient whole genome duplication event about 58–60 Mya and recent event about 13 Mya were take place in soybean [47] but variation in the function of duplicated genes were difficult to understand. The GmSS gene family was also gone through the duplication event and segmental duplication was observed in 92% (12 of 13) GmSS genes (Fig 2).

The Ka/Ks ratio is very important to predict the selection process history of coding region of the genes [55]. The Ka, Ks, and Ka/Ks ratio of the GmSS paralogous members were calculated to investigate the variation in the duplicated GmSS genes. The Ks value was used to estimate the partition of each gene from the paralogous pair. The Ks values (0.031 to 0.11) were observed in all the GmSS paralogous pairs, which fall within the soybean duplication event (Table 3). The six GmSS pairs were duplicated from 2.55 to 9.07 Mya (Table 3). The Ka/Ks ratio was used to determine the selection pressure. The paralogous pairs under purifying selection, positive selection or neutral selection were predicted through Ka/Ks value [56]. The GmSS segmentally duplicated paralogous pairs was under purifying selection with Ka/Ks value <1 (Table 3).

**Table 3:** Ka Ks values and gene duplication of GmSS paralogous gene pairs.

No.	Paralogous	Ka	Ks	Ka/Ks	Time (Mya)	Duplication
1	Glyma16g34290(GmSS9)-Glyma09g29710(GmSS4)	0.01	0.04	0.27	2.99	SD
2	Glyma18g04990(GmSS13)-Glyma11g33240(GmSS12)	0.08	0.11	0.70	9.07	SD
3	Glyma14g39070(GmSS6)-Glyma02g40740(GmSS1)	0.0045	0.04	0.11	3.43	SD
4	Glyma17g05067(GmSS10)-Glyma13g17421(GmSS5)	0.0035	0.05	0.07	4.12	SD
5	Glyma15g20180(GmSS8)-Glyma09g08550(GmSS3)	0.01	0.06	0.18	4.66	SD
6	Glyma19g40041(GmSS11)-Glyma03g37441(GmSS2)	0.008	0.03	0.25	2.55	SD

SD: Segmental duplication.

The protein structure and function were maintained through the preservation of amino acid position during evolutionary process. The selection pressure recognizes the important amino acid, which play an important role in the SS protein interaction. The MEC model was used to calculate the selection pressure in the specific coding sites of GmSS proteins. The deviation in the substitution rate of the coding sites of the amino acids was taken, which used to control the adaptive selectin pressure in the amino acids of GmSS protein (Fig 3). About 1% positive selection was observed in the amino acids of the GmSS protein family through MEC model, while rest of the 99% amino acids was under purifying process (Fig 3), which indicates that GmSS protein family was gone through evolution process under the effect of purifying selection.

**Fig 3:** Selection pressures among SS gene sequences using mechanistic empirical combination (MEC) model of selection online tool. Yellow and brown highlights represent positive selection, gray and white highlights represent neutral selection, and purple highlight represents purifying or negative selection on codons.

Various positive selection sites were found in the SS coding sequence through different tests. The online SLAC and REL tests were used to compute the ω values to figout the evolutionary signals of positive selection. The SS genes in various plant species had strong signal of positive selection. Fifteen amino acids under positive selection in SLAC and eighteen in REL test were detected (Table 4). Confident interval 95% were used in REL test to detect the positive sites through Bayes factor with values > 20. Significance for SLAC test were measured at p-value < 0.2.

**Table 4:** Log likelihood values of positively selected coding sites in SS family genes through different models.

Gene	No. of codons	No. of sequences	SLAC		REL	
SS	942	19	**Coding sites**	**p-value**	**Coding sites**	**ω values**
			**7**	0.02	*7*	0.93
			**83**	0.04	**41**	0.88
			84	0.08	*84*	0.98
			**85**	0.04	*85*	0.93
			112	0.06	*889*	0.98
			135	0.09	*891*	0.98
			208	0.09	*892*	0.97
			222	0.09	*900*	0.98
			254	0.07	*901*	0.98
			258	0.09	*903*	0.98
			312	0.09	*904*	0.98
			**468**	0.05	*905*	0.98
			469	0.06	*910*	0.98
			*608*	0.01	*912*	0.98
			807	0.07	*913*	0.98
					*914*	0.98
					*917*	0.98
					*919*	0.98

In SLAC model, the positively selected sites with probability ≤ 0.01 are italicized while ≤ 0.05 in bold with posterior probability 1.059 while in REL model, the positively selected sites with posterior probability 0.9 are italicized, 0.8–0.89 in bold.

### Protein–protein interaction (PPI) network

GmSS5 protein were analysed in STRING database, number of PPI pairs were found that were interacted with them. We have found a PPI interaction that contains 14 nodes (Fig 4; S1 Table in S1 File). The co-expression was found between sucrose synthase (SS5) and glucose-1-phosphate adenylyltransferase (GLYMA02G47460, GLYMA11G12410, GLYMA06G01380, GLYMA12G04630, GLYMA04G01350) proteins in the PPI network (S1 Table in S1 File). This interaction clearly showed the relation between the protein played vital role in starch synthesis and UDP-glucose and fructose provider for various metabolic pathways.

**Fig 4:** The protein–protein interaction (PPI) network built by STRING database for GmSS5 gene. Line thickness indicates the strength of the interaction. Network nodes denote proteins’ post-transcriptional modifications or splice isoforms, and each node represents all the proteins produced by a single, protein-coding gene locus.

### Phylogenetic analysis and structural investigation of GmSS protein family

Relatively profound evolutionary origin and recent duplication within the gene family was revealed through phylogenetic analysis. The unrooted phylogenetic tree was constructed from the protein sequences of SS genes from *G*. *max*, *A*. *thaliana* and some other plants to examine the evolutionary relationship within the family (Fig 5). Like the previous studies, GmSS genes were also distributed into three classes i.e., class I, class II and class III based on statistical support (Fig 5). It was suggested from the phylogenetic analysis that duplication have increased the SS genes in the classes. Class I contains four GmSS (*GmSS3*, *5*, *8*, *10*) genes and clustered with *AtSS1* and *AtSS2* while class II contains three GmSS (*GmSS2*, *7*, *11*) genes and clustered with *AtSS3* and *AtSS4*. Class III contains large number of GmSS as compare to other two groups that were *GmSS1*, *4*, *6*, *9*, *12* and *13* clustered with *AtSS5* and *AtSS6* (Fig 5). The perceptible diversification within GmSS gene family could involve in distinct function for paralogous regardless of high similarities in their sequences.

**Fig 5:** Phylogenetic tree of soybean SS genes with *AtSS* and other crop plants SS genes. The phylogenetic tree was constructed by MEGA 7.0 using the Neighbour joining method. Bootstrap values in percentage (1000 replicates) are indicated on the nodes. Different classes are highlighted using different colors (Class I in maroon, Class II in blue, and Class III in green).

The variation within the protein family plays an important role to understand its structure and function. The online server (MEME) found the 10 conserved region (motifs) in the GmSS protein sequences with different length and amino acids (Table 5). The six out of ten motifs were found to be representatives of SS gene family through Pfam and SMART tools (Table 5). All the 13 GmSS genes contain all 10 motifs. It was observed that common motif profile was found in similar proteins i.e., GmSS1/6, GmSS4/9, Gmss5/10, GmSS3/8, GmSS2/11 and GmSS12/13 (Fig 6). The differences in the motif composition were also found within the three classes of GmSS family.

**Fig 6:** Protein motifs of soybean SS family. The motifs of soybean SS proteins are shown as colored boxes.

**Table 5:** Conserved motifs in GmSS genes sequences.

No.	Motif	Size	Description
1	GAFVQPALYEAFGLTVVEAMTCGLPTFATCQGGPAEIIVHGVSGFHIDPY	50	Glycosyl transferases group 1
2	YHFSCQFTADLIAMNAADFIITSTYQEIAGSKDTVGQYESHTAFTLPGLY	50	Sucrose synthase
3	FNVVILSPHGYFGQABVLGLPDTGGQVVYILDQVRALENEMLLRIKQQGL	50	Sucrose synthase
4	LZGKPDLIIGNYSDGNLVASLLAHKLGVTQCTIAHALEKTKYPDSDIYWK	50	Sucrose synthase
5	KSKDREEMAEIKKMHDLIEKYNLKGQFRWIAAQTNRYRNGELYRVIADTK	50	No Description
6	EHIGYLKDRSKPIIFSMARLDRVKNJTGLVEWYGKNKRLRELVNLVVVGG	50	No Description
7	RVVHGIBVFDPKFNIVSPGADQSIYFPYT	29	Sucrose synthase
8	ILRVPFRTEKGILRQWISRFDIWPYLETF	29	Sucrose synthase
9	HGDEASDKJVDFFEKCKLDPSHWNKISKAGLQRINEC	37	No Description
10	FEYRFKEWGFERGWGDTAERVKETMQLLLEILZAPDPVTLETFLGRVPMV	50	Sucrose synthase

### Synteny analysis

To understand the evolutionary mechanism of SS gene family in soybean, syntenic analysis was done between *G*. *max* and *A*. *thalina*. Fourteen SS orthologous pairs was found between two studied genomes (Fig 7). Synteny analysis revealed the presence of conserved regions/genes on different soybean chromosomes. All the GmSS genes had the syntenic region in the *A*. *thaliana* genome except *GmSS4* and *GmSS9*. *AtSUS* have evolutionary relationship with multiple GmSS genes like *AtSUS1* have the relationship with four GmSS, *AtSUS4* with three, while *AtSUS2*, *AtSUS3* and *AtSUS5* have relationship with two GmSS genes (Fig 7).

**Fig 7:** Synteny analysis of SS gene pairs between *G*. *max* and *A*. *thaliana*.

### Expression analysis of GmSS genes in different soybean tissues

The expression data of identified GmSS genes in seven different soybean tissues (Seed, Root, Nodule, Stem. Leaf, Flower, and Pod) were retrieved from Pytozome and heatmap was constructed (Fig 8; S2 Table in S1 File). Tissue and organ specific expression of different GmSS genes were observed (Fig 8B). The members of specific class expressed specifically. The class I and class II members highly expressed in all the seven soybean tissues while majority of class III members showed lower expression. However, the class I genes expression was specific to the transport (root, stem) and storage tissues (pod, seed) along with nodules (Fig 8B). The GmSS7 specifically expressed highly only in seed while GmSS13 expressed specifically in root and pod (Fig 8B). It was suggested that the definite tissue or organ expression of a GmSS gene may play vital role in organ development processes. Furthermore, GmSS tissues specific expression will helpful in future investigation of GmSS gene family’s role in biological function of soybean growth and development.

**Fig 8:** Phylogenetic analyses, tissue specific and response to low pH (4.0) expression of *GmSS* genes. **(A)** Phylogenetic tree and nomination of all soybean SS genes (13 in total). The genes are listed according to the chromosomal arrangement, and different classes are highlighted in different colors: Class I in maroon, Class II in blue, and Class III in green. **(B)** The heat map of 13 GmSS genes expression in different tissues was constructed using TBTool software by average linkage with Euclidean distance. Color key represents the relative transcript abundance of the GmSS genes in seven soybean tissues. The FPKM values were log2 transformed and mean centred by genes using the TBTool software. **(C)** The expression level of different GmSS genes in response to low pH stress were retrieved from generated Solexa sequencing libraries, analyzed and represented by constructing the heat map using TBTool software.

In order to explore the roles of GmSS genes during seed development, the expression profiles of GmSS genes were examined during different stages of seed development. The class I member’s expression was downregulated during seed development as compare to control stage (18 DAF), while the expression of class II members gradually increased during seed development at 18, 25, 35, 50 and 55 DAF in DN47 cultivar (S2 Table S1 File). The members of class III did not show much difference in their expression level during different seed development stages and their expression was much lower than the expression of members of other two classes (S2 Table in S1 File).

Tissue specific data from Phytozome indicated that GmSS was expressed in almost all the parts but with some exceptions. However, they have shown the significant positive response against Al^3+^ and low pH [21]. To investigate the mechanism of GmSS genes regulation in response to low pH stress, the Solexa sequencing libraries was extracted from NCBI DEG database. The analysis of Solexa sequencing libraries showed that most of the GmSS genes of class I and GmSS11 of class II were up-regulated in response to low pH (Fig 8C; S3 Table in S1 File). The transcript of up-regulated genes was increased upto 1-fold in response to low pH stress than control (S3 Table in S1 File). Transcriptomic data showed that the expression of the members of class II except for GmSS11 and all the members of class III did not change significantly or had very low FPKM values (S3 Table in S1 File). These results suggest that GmSS class I may have positive role in tolerance of soybean response to low pH.

### Promoter region analysis of GmSS genes

The presence of *cis*-regulatory region in the 1000bp upstream promoter of each GmSS genes was defined through PlantCARE online tool [35]. A variety of cis-acting motifs were found (Fig 9; S4 Table in S1 File). The 39% elements responsive to light, 27% responsive to hormone, 12% responsive environmental stress and to plant growth each was found in the promoter region of 13 GmSS genes (Fig 9). The abscisic acid (ABA), gibberellic acid (GA), auxin, jasmonic acid, salicylic acid and ethylene regulated transcription factors binding sites was also found in the promoter regions. The motifs related to biotic stress like pathogen defense or abiotic stress like heat and low temperature, drought etc was also observed (S4 Table in S1 File). The GmSS members showed different pattern of cis-acting elements in their promoter region. They contain maximum number of ABRE and ERE elements, which showed their response to different hormones.

**Fig 9:** Cis-element analysis in the *GmSS* gene family. PlantCare were used to analyze the region 1500 bp upstream of each of the GmSS genes. The percentage of responsive elements, hormone responsive elements, environmental stress related elements, plant growth responsive elements and site binding responsive elements (except for TATA and CAAT binding sites) in all GmSS genes.

## Discussion

Taking the advantage of whole genome sequencing of many plants, number of SS isozymes encoding genes has been identified previously from different crop plants. There were six SS genes each were reported in model plant *Arabidopsis* and rice, 8, 8, and 15 were in *Gossypium* species i.e *arboretum*, *raimondii* and *hirsutum*, respectively, while 5 SS genes were reported in *Vitis vinifera* that represents the SS genes identificarion in two flowering plants groups i.e monocot and dicot [25]. Recently, eleven SS genes were mentioned in soybean [25] but In this study, we have extracted 13 SS genes from soybean genome through database search that was the 2^nd^ most number of SS genes as compare to previously reported SS genes in different crop plants except for *G*. *hirsutum*. Additionally, exploration of gene family about their evolutionary relationship, gene structure, and expression pattern in different tissues is one of the most imperative step towards complete understanding of molecular mechanism and their possible function involved in various growth processes of soybean.

### Conservation and divergence at evolutionary point of view in GmSS family

Few number of SS encoded enzyme were reported in different plant species [57–60]. The conserved region analysis, chromosomal distribution, duplication events, positive selection, gene structure, phylogenetic and expression analysis of gene family facilitate the researchers to examine their possible function and ancestor relationship among identified and unidentified family members. The similarity/identity in the gene sequence were found conserved among homologous genes within the family and their analysis can give an evidence to expose the evolutionary background of the definite gene family. The present gene family analysis revealed that the predicted molecular characteristics of the GmSS proteins were in account with the previously characterized SS from different plant species.

However, the successive chromosomal reshuffling and duplication event have differentially formed the SS protein family in soybean genome. Further, analysis was done to investigate that whether GmSS gene structure models were related to their phylogenetic relationship. The unrooted phylogenetic tree clustered the 13 GmSS genes into three different classes that indicates the link between GmSS protein structure and evolutionary history (Fig 8A). The maintenance and deviation among GmSS genes structure, expend the number of genes within the family that leads in conservation or differences in their functions. Generally, gain/loss of exon-intron, exonization/pseudo-exonization and insertion/deletion were the three main mechanism that had the role in the expansion of gene family [61]. The GmSS also distributed into three classes that was consistent with the previously distribution of SS family members [59, 62]. It was suggested that expansion of class III (GmSS12/GmSS13) members was the earliest through evolutionary branch analysis. So the GmSS12/GmSS13 had the oldest evolutionary history than other members that ultimately leads towards their complex structure (Table 3). The tandem and segmental duplication events increased the gene numbers in a family [63] that leads to their functional redundancy, sub-functionalization and neo-functinalization [25]. The duplicated gene pairs in GmSS gene family shares high level of similarity and identity at amino acid level like GmSS5–GmSS10 had 99.63% similarity and 98.88% identity at sequence level with same gene length, protein properties, gene structure but little variation in gene expression in flower and pod (Tables 1 and 2; Fig 8). Furthermore, the paralogous GmSS gene pair had firm phylogenetic relationship among different plant SS gene families and within soybean SS genes (Figs 5 and 8A).

Polyploidy play an important role in the adaptation of flowering plants into new environmental condition during their evolutionary phase [64]. In soybean, polyploidy was an important point, hence the duplication arising from the doubling of SS genes in numbers. Even duplication is affected by polyploidy; due to segment duplication, the SS gene is also increased. Segment duplication plays an important role in the evolution of plants, because the number of flowering plants diploid and polyploid and maintained the duplicated chromosome within the plant genome [65]. We found that 12 of the 13 genes caused the amplification of the SS gene because they are related to the segmental duplication and are significantly affected by these duplications. Due to the tetraploid nature of soybeans, compared with other crops, the segmented duplication of the SS gene found in soybeans, is the second largest in number. The genome size of the soybean is increased due to duplication event, causing the number of chromosomes to increase from 10 to 20. Therefore, the extension of the GmSS gene is significantly attributed to genomic duplication. In addition, the diversity of GmSS genes related to the quality, structure and function of the SS family may be affected by the duplication and expansion of this gene family.

Molecular structure and phylogenetic analysis of previous SS gene family studies distributed the genes in to SS1, SSA and New Group [22, 66]. Number of studies substantiated the SS genes distribution and groups were named as Class I, Class II and Class III [25, 50, 53]. The Class I group of SS gene family in number of plant species further divided into monocot and eudicot subclasses that were distinct from each other in phylogenetic tree. Whereas, Class II and Class III were also divided into mix group 1 and mix group 2 because they also contains the monocot and eudicot [25, 57].

It was revealed from the phylogenetic tree of 13 GmSS, 6 AtSS and 12 from other plant species that each class contains atleast three GmSS members in each class. Among the 13 GmSS genes, GmSS5/10, GmSS3/8 clustered in Class I, GmSS2/11 in Class II, while GmSS7 alone clustered into one branch in Class II, GmSS1/6 and GmSS12/13 clustered closely together in one branch of Class III, whereas GmSS4/9 cluster together in another branch of Class III (Fig 5). The fall of GmSS in separate branch showed their variation in the structure and may perform different function within the metabolic functions in soybean. All the GmSS genes were appeared separately from AtSS genes except for GmSS that closely related with AtSS4 (Fig 5). It indicates that the duplication event in soybean SS take place after monocot-eudicot separation but earlier than Glycine/Arabidopsis divergence. The two members of leguminosae family i.e soybean and pea, had a close evolutionary relationship. The paralogous pair GmSS3/8 closely related with PsSS3 and GmSS2/11 with PsSS2 suggesting their relation between two plant of the same family. However, GmSS did not have any close clustering with other crops SS like *Z*. *mays*, *T*. *aestivum*, *P*. *trichocarapa* and *C*. *unshiu* (Fig 5). Therefore, the duplication event in GmSS12/13 was observed more earliest than other GmSS while the recent duplication event was noted in GmSS2/11 (Table 3). The positive selection may had a vital impact on the evolution of the gene family. The process of selection can reveal the important amino acids within the gene family.

Positive selection analysis shows that each branch of the phylogenetic tree has been studied, and there are several codon sites in the positive selection of the SS gene family (Fig 3). Rapid gene evolution and branch length are the main components of positive selection, and related genes are frequently modified to enter positive selection (Fig 9; [67]). We found through MEC that only 1% of SS amino acids are in a positive selection state, while the remaining amino acids are in the purification process. The dN/dS ratio of Glycine-Cytosine subjective genes increases and may produce false positive amino acids in the branch site model of positive selection [68]. In addition, the GmSS genes were observed to understand the evolutionary dynamics and consequences. Based on Ka/Ks values, a large number of genes are under purifying selection, showing a strong gene duplication effect (Table 3). Next, observe the difference in expression between the six duplicated GmSS gene pairs. The same expression pattern of duplicated genes was found as the original gene, but with slight variations in expression (Fig 6). More observations revealed the existence of different expression patterns in duplicated genes, suggesting new functional evolutions after duplication.

This was done to examine that whether the various studied plant species present the phylogenetic relationship and showed the selection pressure or give some evolutionary evidence of their native periodic positive selection. When the branches of phylogenetic tree were examined, the sequences of examined genes showed the various coding sites under positive selection. The SLAC and REL found 15 and 18 coding sites, respectively, that was under positive selection in SS gene family (Table 4). The positively detected sites within the sequence take major contribution in the divergence of gene function among different plant species. Variation in the functional and expression of mutated gene is predicted to encourage the maintenance of the gene sequence [69, 70]. The divergence in the mutated genes due to positive selection and constraints in the subsequent selection, leads to their functional variation. However, the variation in the coding sites that leads to reduce the gene function are removed through negative selection and variation in the coding region that increased and stabilize the gene function are preserve through positive selection [71].

### GmSS gene family role in soybean growth and development

Gene duplication varies the function of the protein that ultimately change the expression and protein property and recognized main evolutionary driver that can improve the plant to fit in the new environment [72]. The genes involved in the physiological process of the plants can be predicted through expression profile analysis of the respective gene. Although, the detailed expression analysis of SS genes were previously mentioned in different plant species [25, 50, 73], and here we mentioned the expression profile of GmSS in different soybean tissues and at different seed developmental stages using an expression atlas of *G*. *max* (Fig 8; S2 Table in S1 File). The high expression of *GmSS5*, *GmSS10* and *GmSS11* gene in specific soybean tissues that probably imitate their role in a common metabolic and/or developmental process. High expression of *GmSS5* and *GmSS10* in nodule, seed and pod along with stem suggested that these genes had vital role in sugar regulation, accumulation and in soybean seed and transport in soybean stem. The high expression of *GmSS11* in flower suggested its role in energy supply within reproductive organ to support the development process from bud to flower (Fig 8; S2 Table in S1 File). However, the spatial-temporal expression of SS genes in other plants like during the early stages of apple fruit development, the SS genes expression was very high. But the SS genes down-regulated due to cell expansion and fruit increased in size [74]. Similarly, the *CitSus* genes also showed variation in their expression related to their function and organ. The *CitSus1* and *CitSus2* were highly expressed in fruit juice sac while *CitSus3* and *CitSus4* in immature leaves and *CitSus5*, *CitSus6* were expressed in both fruit juice sac as well as in immature leaves. But the *CitSus5* expression significantly increased and *CitSus6* decreased in fruit juice sac during fruit development. *NtSus2* and *NtSus3* had high expression during tobacco leave development and played vital role in sucrose metabolism [62]. Likewise, the *GrSUS1*, *GrSUS2*, and *GrSUS3* expressed significantly higher and frequently changed during fiber development in *Gossypium* species [53]. The redundant or low expression of *VvSS1*, *VvSS2* and *VvSS3* was observed during *V*. *vinifera* growth and development [25]. But other VvSS genes highly expressed in different tissues like seed-PFS, tendril and played important function [25]. Similar type of variation in GmSS genes expression level during seed development was observed (S2 Table in S1 File). *GmSS3* and *GmSS8* had significantly higher expression levels and underwent significant changes in expression during seed development. The members of the Class III were not expressed, or were expressed at low levels, suggesting their redundant function in the normal development of soybean seed (S2 Table in S1 File). It was suggested that GmSS genes performed their role diversely and overlapped partially. However, cell division and vascular tissues differentiation in leaves had adversely affected by sucrose [25] but the overall transcript level comparison of GmSS family members in each tissues revealed their predominant role of GmSS genes of Class I and GmSS11 in soybean growth and development (Fig 8).

The plant rhizophere toxicity in the acidic soil was due to accumulation of H^+^ and Al^3+^ that ultimately cause the oxidative stress, lipid composition changes, membrane disintegrity, mitochondria dysfunction, protein denaturation, DNA damage and cell-cycle blockage in the plant organs especially in roots [75, 76]. There was number of mechanism involved through which a plant response to Al^3+^ stress. We have found five GmSS genes that up-regulated upto 30-fold in response to Al^3+^ and low pH stress, suggesting their putative role against these two stresses. However, Al stress alone suppressed the expression of SuS genes in barley but significantly up-regulated their expression in combine stress of Al and PEG at low pH (4.0) [21]. SuS genes along-with KS-DHN had important role in plant adaptation in response to drought at cellular level [77, 78] suggesting that it may be due to the induction of ABA that maintain the root hair growth [21]. ABA improves the root ability to uptake the sucrose efficiently in sugar beet [79] while the *abi8* Arabidopsis mutant plants showed significantly down-regulation of sucrose synthase genes [80]. Hence, it was suggested that Al may inhibit the root elongation under drought stress through the deactivation of ABA-dependent drought induced gene regulation [21]. It was reported that Al interfere with different plant regulatory mechanism that were involved in ABA signal transduction and crosstalk with other drought stress related important hormones [81].

This study was evaluated by examining the putative function of promoter sequence. Our bioinformatic study demonstrated the presence of important *cis*-acting regions in upstream of the GmSS gene that regulate hormones and stress responsive elements. The composition of the regulatory elements differs in GmSS in response to different stimuli. The GmSS promoter region also contains a wide range of elements related to light, hormone, biological and abiotic. GmSS promoter conserved the regulatory elements just like other model plants.

## Conclusions

The findings of the present study can be used for future crop improvement program for cloning, characterization and detailed investigation of SS genes in soybean. The role of GmSS genes in *G*. *max* growth, sucrose metabolism and response to different factors can be clarified in further studies that can explore the potential function of the identified candidate GmSS genes with enhanced productivity.

## Supporting information

S1 File Supporting files of the expression analysis between sucrose synthase and glucose-1-phosphate adenylyltransferase proteins. (XLSX)

## References

[1] SchmalstigJG, HitzWD. Contributions of sucrose synthase and invertase to the metabolism of sucrose in developing leaves: estimation by alternate substrate utilization. Plant Physiology. 1987;85(2):407–12. doi: 10.1104/pp.85.2.407 16665711PMC1054269

[2] GeigenbergerP, StittM. Sucrose synthase catalyses a readily reversible reaction in vivo in developing potato tubers and other plant tissues. Planta. 1993;189(3):329–39. doi: 10.1007/BF00194429 24178489

[3] KleczkowskiLA, KunzS, WilczynskaM. Mechanisms of UDP-glucose synthesis in plants. Crit Rev Plant Sci. 2010;29(4):191–203.

[4] AlbrechtG, MustrophA. Localization of sucrose synthase in wheat roots: increased *in situ* activity of sucrose synthase correlates with cell wall thickening by cellulose deposition under hypoxia. Planta. 2003;217(2):252–60. doi: 10.1007/s00425-003-0995-6 12783333

[5] FujiiS, HayashiT, MizunoK. Sucrose synthase is an integral component of the cellulose synthesis machinery. Plant and Cell Physiology. 2010;51(2):294–301. doi: 10.1093/pcp/pcp190 20056592

[6] NolteKD, HendrixDL, RadinJW, KochKE. Sucrose synthase localization during initiation of seed development and trichome differentiation in cotton ovules. Plant Physiology. 1995;109(4):1285–93. doi: 10.1104/pp.109.4.1285 12228669PMC157661

[7] BarrattDP, BarberL, KrugerNJ, SmithAM, WangTL, MartinC. Multiple, distinct isoforms of sucrose synthase in pea. Plant Physiology. 2001;127(2):655–64. 11598239PMC125100

[8] FuH, ParkWD. Sink-and vascular-associated sucrose synthase functions are encoded by different gene classes in potato. The Plant Cell. 1995;7(9):1369–85. doi: 10.1105/tpc.7.9.1369 8589622PMC160958

[9] TangG-Q, LüscherM, SturmA. Antisense repression of vacuolar and cell wall invertase in transgenic carrot alters early plant development and sucrose partitioning. The Plant Cell. 1999;11(2):177–89. doi: 10.1105/tpc.11.2.177 9927637PMC144160

[10] ZrennerR, SalanoubatM, WillmitzerL, SonnewaldU. Evidence of the crucial role of sucrose synthase for sink strength using transgenic potato plants (*Solanum tuberosum* L.). The Plant Journal. 1995;7(1):97–107. doi: 10.1046/j.1365-313x.1995.07010097.x 7894514

[11] KlotzKL, FingerFL, ShelverWL. Characterization of two sucrose synthase isoforms in sugarbeet root. Plant Physiol Biochem. 2003;41(2):107–15.

[12] SunJ, LobodaT, SungS-JS, BlackCCJr. Sucrose synthase in wild tomato, *Lycopersicon chmielewskii*, and tomato fruit sink strength. Plant Physiology. 1992;98(3):1163–9. doi: 10.1104/pp.98.3.1163 16668741PMC1080322

[13] BieniawskaZ, Paul BarrattD, GarlickAP, TholeV, KrugerNJ, MartinC, et al. Analysis of the sucrose synthase gene family in Arabidopsis. The Plant Journal. 2007;49(5):810–28. doi: 10.1111/j.1365-313X.2006.03011.x 17257168

[14] HaradaT, SatohS, YoshiokaT, IshizawaK. Expression of sucrose synthase genes involved in enhanced elongation of pondweed (*Potamogeton distinctus*) turions under anoxia. Ann Bot. 2005;96(4):683–92. doi: 10.1093/aob/mci220 16033779PMC4247035

[15] BaierMC, KeckM, GoݶddeV, NiehausK, KuݶsterH, HohnjecN. Knockdown of the symbiotic sucrose synthase *MtSucS1* affects arbuscule maturation and maintenance in mycorrhizal roots of *Medicago truncatula*. Plant Physiology. 2010;152(2):1000–14. doi: 10.1104/pp.109.149898 20007443PMC2815868

[16] HohnjecN, PerlickAM, PühlerA, KüsterH. The *Medicago truncatula* sucrose synthase gene *MtSucS1* is activated both in the infected region of root nodules and in the cortex of roots colonized by arbuscular mycorrhizal fungi. Mol Plant-Microbe Interact. 2003;16(10):903–15. doi: 10.1094/MPMI.2003.16.10.903 14558692

[17] CarlsonSJ, ChoureyPS, HelentjarisT, DattaR. Gene expression studies on developing kernels of maize sucrose synthase (SuSy) mutants show evidence for a third SuSy gene. Plant Mol Biol. 2002;49(1):15–29. doi: 10.1023/a:1014457901992 12008896

[18] ChoureyP, TaliercioE, CarlsonS, RuanY-L. Genetic evidence that the two isozymes of sucrose synthase present in developing maize endosperm are critical, one for cell wall integrity and the other for starch biosynthesis. Molecular and General Genetics MGG. 1998;259(1):88–96. doi: 10.1007/s004380050792 9738884

[19] LiuJ, LiY, WangW, GaiJ, LiY. Genome-wide analysis of MATE transporters and expression patterns of a subgroup of MATE genes in response to aluminum toxicity in soybean. BMC Genomics. 2016;17(1):1–15.2696851810.1186/s12864-016-2559-8PMC4788864

[20] ChandranD, SharopovaN, VandenBoschKA, GarvinDF, SamacDA. Physiological and molecular characterization of aluminum resistance in *Medicago truncatula*. BMC Plant Biology. 2008;8(1):1–17. doi: 10.1186/1471-2229-8-89 18713465PMC2533010

[21] AhmedIM, NadiraUA, CaoF, HeX, ZhangG, WuF. Physiological and molecular analysis on root growth associated with the tolerance to aluminum and drought individual and combined in Tibetan wild and cultivated barley. Planta. 2016;243(4):973–85. doi: 10.1007/s00425-015-2442-x 26748913

[22] HorstI, WelhamT, KellyS, KanekoT, SatoS, TabataS, et al. TILLING mutants of *Lotus japonicus* reveal that nitrogen assimilation and fixation can occur in the absence of nodule-enhanced sucrose synthase. Plant Physiology. 2007;144(2):806–20. doi: 10.1104/pp.107.097063 17468221PMC1914161

[23] HuangJ-W, ChenJ-T, YuW-P, ShyurL-F, WangA-Y, SungH-Y, et al. Complete structures of three rice sucrose synthase isogenes and differential regulation of their expressions. Biosci, Biotechnol, Biochem. 1996;60(2):233–9. doi: 10.1271/bbb.60.233 9063969

[24] WangA-Y, KaoM-H, YangW-H, SayionY, LiuL-F, LeeP-D, et al. Differentially and developmentally regulated expression of three rice sucrose synthase genes. Plant and Cell Physiology. 1999;40(8):800–7. doi: 10.1093/oxfordjournals.pcp.a029608 10555303

[25] ZhuX, WangM, LiX, JiuS, WangC, FangJ. Genome-wide analysis of the sucrose synthase gene family in grape (*Vitis vinifera*): structure, evolution, and expression profiles. Genes. 2017;8(4):111.10.3390/genes8040111PMC540685828350372

[26] GoodsteinDM, ShuS, HowsonR, NeupaneR, HayesRD, FazoJ, et al. Phytozome: a comparative platform for green plant genomics. Nucleic Acids Research. 2012;40(D1):D1178–D86. doi: 10.1093/nar/gkr944 22110026PMC3245001

[27] JoshiT, FitzpatrickMR, ChenS, LiuY, ZhangH, EndacottRZ, et al. Soybean knowledge base (SoyKB): a web resource for integration of soybean translational genomics and molecular breeding. Nucleic Acids Research. 2014;42(D1):D1245–D52. doi: 10.1093/nar/gkt905 24136998PMC3965117

[28] Marchler-BauerA, BoY, HanL, HeJ, LanczyckiCJ, LuS, et al. CDD/SPARCLE: functional classification of proteins via subfamily domain architectures. Nucleic Acids Research. 2017;45(D1):D200–D3. doi: 10.1093/nar/gkw1129 27899674PMC5210587

[29] GasteigerE, GattikerA, HooglandC, IvanyiI, AppelRD, BairochA. ExPASy: the proteomics server for in-depth protein knowledge and analysis. Nucleic Acids Research. 2003;31(13):3784–8. doi: 10.1093/nar/gkg563 12824418PMC168970

[30] WolfeD, DudekS, RitchieMD, PendergrassSA. Visualizing genomic information across chromosomes with PhenoGram. BioData Mining. 2013;6(1):1–12. doi: 10.1186/1756-0381-6-1 24131735PMC4015356

[31] KumarS, StecherG, TamuraK. MEGA7: molecular evolutionary genetics analysis version 7.0 for bigger datasets. Molecular Biology and Evolution. 2016;33(7):1870–4. doi: 10.1093/molbev/msw054 27004904PMC8210823

[32] JabbirF, IrfanM, MustafaG, AhmadHI. Bioinformatics approaches to explore the phylogeny and role of BRCA1 in breast cancer. Critical Reviews™ in Eukaryotic Gene Expression. 2019;29(6). doi: 10.1615/CritRevEukaryotGeneExpr.2019030785 32422010

[33] BaileyTL, WilliamsN, MislehC, LiWW. MEME: discovering and analyzing DNA and protein sequence motifs. Nucleic Acids Research. 2006;34(suppl_2):W369–W73. doi: 10.1093/nar/gkl198 16845028PMC1538909

[34] PuntaM, CoggillPC, EberhardtRY, MistryJ, TateJ, BoursnellC, et al. The Pfam protein families database. Nucleic Acids Research. 2012;40(D1):D290–D301. doi: 10.1093/nar/gkr1065 22127870PMC3245129

[35] LescotM, DéhaisP, ThijsG, MarchalK, MoreauY, Van de PeerY, et al. PlantCARE, a database of plant cis-acting regulatory elements and a portal to tools for in silico analysis of promoter sequences. Nucleic Acids Research. 2002;30(1):325–7. doi: 10.1093/nar/30.1.325 11752327PMC99092

[36] LynchM, ConeryJS. The evolutionary fate and consequences of duplicate genes. Science. 2000;290(5494):1151–5. doi: 10.1126/science.290.5494.1151 11073452

[37] Doron-FaigenboimA, PupkoT. A combined empirical and mechanistic codon model. Molecular Biology and Evolution. 2007;24(2):388–97. doi: 10.1093/molbev/msl175 17110464

[38] AhmadHI, LiuG, JiangX, LiuC, ChongY, HuarongH. Adaptive molecular evolution of MC 1R gene reveals the evidence for positive diversifying selection in indigenous goat populations. Ecology and evolution. 2017;7(14):5170–80. doi: 10.1002/ece3.2919 28770057PMC5528238

[39] YangZ. PAML: a program package for phylogenetic analysis by maximum likelihood. Comput Appl Biosci. 1997;13(5):555–6. doi: 10.1093/bioinformatics/13.5.555 9367129

[40] AhmadMJ, AhmadHI, AdeelMM, LiangA, HuaG, MurtazaS, et al. Evolutionary analysis of makorin ring finger protein 3 reveals positive selection in mammals. Evolutionary Bioinformatics. 2019;15:1176934319834612. doi: 10.1177/1176934319834612 31024214PMC6472170

[41] PondSLK, FrostSD. Datamonkey: rapid detection of selective pressure on individual sites of codon alignments. Bioinformatics. 2005;21(10):2531–3. doi: 10.1093/bioinformatics/bti320 15713735

[42] AhmadHI, AsifAR, AhmadMJ, JabbirF, AdnanM, AhmedS, et al. Adaptive evolution of peptidoglycan recognition protein family regulates the innate signaling against microbial pathogens in vertebrates. Microbial Pathogenesis. 2020;147:104361. doi: 10.1016/j.micpath.2020.104361 32622926

[43] AhmadHI, ZhouJ, AhmadMJ, AfzalG, JiangH, ZhangX, et al. Adaptive selection in the evolution of programmed cell death-1 and its ligands in vertebrates. Aging (Albany NY). 2020;12(4):3516. doi: 10.18632/aging.102827 32045365PMC7066927

[44] ChenC, ChenH, ZhangY, ThomasHR, FrankMH, HeY, et al. TBtools: an integrative toolkit developed for interactive analyses of big biological data. Molecular Plant. 2020;13(8):1194–202. doi: 10.1016/j.molp.2020.06.009 32585190

[45] FranceschiniA, SzklarczykD, FrankildS, KuhnM, SimonovicM, RothA, et al. STRING v9. 1: protein-protein interaction networks, with increased coverage and integration. Nucleic Acids Research. 2012;41(D1):D808–D15. doi: 10.1093/nar/gks1094 23203871PMC3531103

[46] AhmadHI, AhmadMJ, AdeelMM, AsifAR, DuX. Positive selection drives the evolution of endocrine regulatory bone morphogenetic protein system in mammals. Oncotarget. 2018;9(26):18435. doi: 10.18632/oncotarget.24240 29719616PMC5915083

[47] SchmutzJ, CannonSB, SchlueterJ, MaJ, MitrosT, NelsonW, et al. Genome sequence of the palaeopolyploid soybean. Nature. 2010;463(7278):178–83. doi: 10.1038/nature08670 20075913

[48] SongB, AnL, HanY, GaoH, RenH, ZhaoX, et al. Transcriptome profile of near-isogenic soybean lines for *β*-conglycinin *α*-subunit deficiency during seed maturation. PLoS One. 2016;11(8):e0159723. doi: 10.1371/journal.pone.0159723 27532666PMC4988716

[49] ChenQ, WuW, ZhaoT, TanW, TianJ, LiangC. Complex Gene Regulation Underlying Mineral Nutrient Homeostasis in Soybean Root Response to Acidity Stress. Genes. 2019;10(5):402. doi: 10.3390/genes10050402 31137896PMC6563148

[50] ChenA, HeS, LiF, LiZ, DingM, LiuQ, et al. Analyses of the sucrose synthase gene family in cotton: structure, phylogeny and expression patterns. BMC Plant Biology. 2012;12(1):1–17. doi: 10.1186/1471-2229-12-85 22694895PMC3505178

[51] HardinSC, HuberSC. Proteasome activity and the post-translational control of sucrose synthase stability in maize leaves. Plant Physiol Biochem. 2004;42(3):197–208. doi: 10.1016/j.plaphy.2003.12.004 15051043

[52] HuberSC, HuberJL, LiaoP-C, GageDA, McMichaelRWJr, ChoureyPS, et al. Phosphorylation of serine-15 of maize leaf sucrose synthase (occurrence in vivo and possible regulatory significance). Plant Physiology. 1996;112(2):793–802. doi: 10.1104/pp.112.2.793 8883390PMC158004

[53] ZouC, LuC, ShangH, JingX, ChengH, ZhangY, et al. Genome‐W ide Analysis of the Sus Gene Family in Cotton. Journal of Integrative Plant Biology. 2013;55(7):643–53. doi: 10.1111/jipb.12068 23691964

[54] KongH, LandherrLL, FrohlichMW, Leebens‐MackJ, MaH, DePamphilisCW. Patterns of gene duplication in the plant SKP1 gene family in angiosperms: evidence for multiple mechanisms of rapid gene birth. The Plant Journal. 2007;50(5):873–85. doi: 10.1111/j.1365-313X.2007.03097.x 17470057

[55] LiW-H, GojoboriT, NeiM. Pseudogenes as a paradigm of neutral evolution. Nature. 1981;292(5820):237–9. doi: 10.1038/292237a0 7254315

[56] JureticN, HoenDR, HuynhML, HarrisonPM, BureauTE. The evolutionary fate of MULE-mediated duplications of host gene fragments in rice. Genome Res. 2005;15(9):1292–7. doi: 10.1101/gr.4064205 16140995PMC1199544

[57] AnX, ChenZ, WangJ, YeM, JiL, WangJ, et al. Identification and characterization of the Populus sucrose synthase gene family. Gene. 2014;539(1):58–67. doi: 10.1016/j.gene.2014.01.062 24508272

[58] VisionTJ, BrownDG, TanksleySD. The origins of genomic duplications in Arabidopsis. Science. 2000;290(5499):2114–7. doi: 10.1126/science.290.5499.2114 11118139

[59] WangZ, WeiP, WuM, XuY, LiF, LuoZ, et al. Analysis of the sucrose synthase gene family in tobacco: structure, phylogeny, and expression patterns. Planta. 2015;242(1):153–66. doi: 10.1007/s00425-015-2297-1 25893870PMC4471321

[60] ZourelidouM, De Torres‐ZabalaM, SmithC, BevanMW. Storekeeper defines a new class of plant‐specific DNA‐binding proteins and is a putative regulator of patatin expression. The Plant Journal. 2002;30(4):489–97. doi: 10.1046/j.1365-313x.2002.01302.x 12028578

[61] XuS-M, BrillE, LlewellynDJ, FurbankRT, RuanY-L. Overexpression of a potato sucrose synthase gene in cotton accelerates leaf expansion, reduces seed abortion, and enhances fiber production. Molecular Plant. 2012;5(2):430–41. doi: 10.1093/mp/ssr090 22115917

[62] IslamMZ, HuX-M, JinL-F, LiuY-Z, PengS-A. Genome-wide identification and expression profile analysis of citrus sucrose synthase genes: investigation of possible roles in the regulation of sugar accumulation. PLoS One. 2014;9(11):e113623. doi: 10.1371/journal.pone.0113623 25420091PMC4242728

[63] CannonSB, MitraA, BaumgartenA, YoungND, MayG. The roles of segmental and tandem gene duplication in the evolution of large gene families in *Arabidopsis thaliana*. BMC Plant Biology. 2004;4(1):1–21. doi: 10.1186/1471-2229-4-10 15171794PMC446195

[64] RamseyJ, SchemskeDW. Pathways, mechanisms, and rates of polyploid formation in flowering plants. Annu Rev Ecol Syst. 1998;29(1):467–501.

[65] CannonSB, KozikA, ChanB, MichelmoreR, YoungND. DiagHunter and GenoPix2D: programs for genomic comparisons, large-scale homology discovery and visualization. Genome Biology. 2003;4(10):1–8. doi: 10.1186/gb-2003-4-10-r68 14519203PMC328457

[66] HiroseT, ScofieldGN, TeraoT. An expression analysis profile for the entire sucrose synthase gene family in rice. Plant Sci. 2008;174(5):534–43.

[67] MeslinC, MugnierS, CallebautI, LaurinM, PascalG, PouponA, et al. Evolution of genes involved in gamete interaction: evidence for positive selection, duplications and losses in vertebrates. PLoS One. 2012:e44548. doi: 10.1371/journal.pone.0044548 22957080PMC3434135

[68] RatnakumarA, MoussetS, GléminS, BerglundJ, GaltierN, DuretL, et al. Detecting positive selection within genomes: the problem of biased gene conversion. Philosophical Transactions of the Royal Society B: Biological Sciences. 2010;365(1552):2571–80. doi: 10.1098/rstb.2010.0007 20643747PMC2935097

[69] ForceA, LynchM, PickettFB, AmoresA, Yan Y-l, Postlethwait J. Preservation of duplicate genes by complementary, degenerative mutations. Genetics. 1999;151(4):1531–45. doi: 10.1093/genetics/151.4.1531 10101175PMC1460548

[70] SémonM, WolfeKH. Consequences of genome duplication. Current opinion in genetics & development. 2007;17(6):505–12. doi: 10.1016/j.gde.2007.09.007 18006297

[71] FettermanCD, RannalaB, WalterMA. Identification and analysis of evolutionary selection pressures acting at the molecular level in five forkhead subfamilies. BMC evolutionary biology. 2008;8(1):261. doi: 10.1186/1471-2148-8-261 18816404PMC2570691

[72] FlagelLE, WendelJF. Gene duplication and evolutionary novelty in plants. New Phytol. 2009;183(3):557–64. doi: 10.1111/j.1469-8137.2009.02923.x 19555435

[73] XiaoX, TangC, FangY, YangM, ZhouB, QiJ, et al. Structure and expression profile of the sucrose synthase gene family in the rubber tree: indicative of roles in stress response and sucrose utilization in the laticifers. The FEBS Journal. 2014;281(1):291–305. doi: 10.1111/febs.12595 24279382

[74] LiM, FengF, ChengL. Expression patterns of genes involved in sugar metabolism and accumulation during apple fruit development. PLoS One. 2012;7(3):e33055. doi: 10.1371/journal.pone.0033055 22412983PMC3296772

[75] DelhaizeE, MaJF, RyanPR. Transcriptional regulation of aluminium tolerance genes. Trends Plant Sci. 2012;17(6):341–8. doi: 10.1016/j.tplants.2012.02.008 22459757

[76] WangJ, HouQ, LiP, YangL, SunX, BeneditoVA, et al. Diverse functions of multidrug and toxin extrusion (MATE) transporters in citric acid efflux and metal homeostasis in *Medicago truncatula*. The Plant Journal. 2017;90(1):79–95. doi: 10.1111/tpj.13471 28052433

[77] BartelsD, SunkarR. Drought and salt tolerance in plants. Crit Rev Plant Sci. 2005;24(1):23–58.

[78] YangZB, EtichaD, RotterB, RaoIM, HorstWJ. Physiological and molecular analysis of polyethylene glycol‐induced reduction of aluminium accumulation in the root tips of common bean (*Phaseolus vulgaris*). New Phytol. 2011;192(1):99–113. doi: 10.1111/j.1469-8137.2011.03784.x 21668875

[79] SaftnerRA, WyseRE. Effect of plant hormones on sucrose uptake by sugar beet root tissue discs. Plant Physiology. 1984;74(4):951–5. doi: 10.1104/pp.74.4.951 16663540PMC1066799

[80] Brocard-GiffordI, LynchTJ, GarciaME, MalhotraB, FinkelsteinRR. The *Arabidopsis thaliana* ABSCISIC ACID-INSENSITIVE8 locus encodes a novel protein mediating abscisic acid and sugar responses essential for growth. The Plant Cell. 2004;16(2):406–21. doi: 10.1105/tpc.018077 14742875PMC341913

[81] YangZ-B, EtichaD, AlbaceteA, RaoIM, RoitschT, HorstWJ. Physiological and molecular analysis of the interaction between aluminium toxicity and drought stress in common bean (*Phaseolus vulgaris*). Journal of Experimental Botany. 2012;63(8):3109–25. doi: 10.1093/jxb/ers038 22371077PMC3350927

